# Morphological Evolution of Pit-Patterned Si(001) Substrates Driven by Surface-Energy Reduction

**DOI:** 10.1186/s11671-017-2320-5

**Published:** 2017-09-29

**Authors:** Marco Salvalaglio, Rainer Backofen, Axel Voigt, Francesco Montalenti

**Affiliations:** 1 Institute of Scientific Computing, Technische Universität Dresden, Dresden, 01062 Germany; 2 0000 0001 0142 678 IHP, Im Technologiepark 25, Frankfurt (Oder), 15236 Germany; 3 Dresden Center for Computational Materials Science (DCMS), Dresden, 01062 Germany; 4 L-NESS and Department of Materials Science, Università di Milano-Bicocca, via R. Cozzi 55, Milano, I-20126 Italy

**Keywords:** Epitaxy, Silicon, Surface diffusion, Phase field, Surface energy

## Abstract

Lateral ordering of heteroepitaxial islands can be conveniently achieved by suitable pit-patterning of the substrate prior to deposition. Controlling shape, orientation, and size of the pits is not trivial as, being metastable, they can significantly evolve during deposition/annealing. In this paper, we exploit a continuum model to explore the typical metastable pit morphologies that can be expected on Si(001), depending on the initial depth/shape. Evolution is predicted using a surface-diffusion model, formulated in a phase-field framework, and tackling surface-energy anisotropy. Results are shown to nicely reproduce typical metastable shapes reported in the literature. Moreover, long time scale evolutions of pit profiles with different depths are found to follow a similar kinetic pathway. The model is also exploited to treat the case of heteroepitaxial growth involving two materials characterized by different facets in their equilibrium Wulff’s shape. This can lead to significant changes in morphologies, such as a rotation of the pit during deposition as evidenced in Ge/Si experiments.

## Background

Lattice-mismatched heteroepitaxy of several semiconductors (such as Ge/Si or InGaAs/GaAs) can lead to the formation of 3D islands, following the Stranski-Krastanow (SK) growth mode. While the possibility to obtain such dots by pure self-assembly [1, 2] is particularly appealing and generated widespread interest, it was soon realized that random nucleation could severely hinder applications, along with dispersion in size and shape.

Decades of research led to the development of a wide variety of methods to drive heteroepitaxial growth towards the formation of ordered structures [3–7]. Among them, the usage of pit-patterned substrates has been demonstrated to be one of the most versatile methods in order to achieve both high ordering and size control of heteroepitaxial islands [8–15].

Pit-patterned substrates are usually fabricated by means of methods such as nanoimprint lithography [16–18], e-beam lithography [13, 14] combined with reactive ion etching (RIE) [19, 20] or wet chemical etching [21, 22], and nanoindentation [23, 24], i.e., by top-down approaches. With these methods, ordered patterns of pits are designed with high precision and, under proper growth conditions [14, 25], lead to almost perfect lateral ordering.

As the actual shape of pits does influence the energy of the system and, more in general, island nucleation [26, 27], it is crucial to control their morphology. This is not trivial: after all, pits are just holes drilled into the substrate. Thus, at sufficiently high temperatures, capillarity [28] is expected to produce a morphological evolution, eventually leading to full healing. Actually, annealing processes or further deposition of the substrate material following the initial pit formation are often used in order to achieve reproducible, long-lived metastable shapes [8, 26]. Notice that even once a pit is stabilized in shape, further evolution can be driven during actual heteroepitaxy [29, 30].

In this work, we aim at describing the evolution of pit-patterned substrates driven by surface energy reduction via surface diffusion. We adopt a suitable phase-field approach [31], allowing for the simulation of length and time scales compatible with the experimental ones [32]. The model has been already adopted to account for diffusion-limited kinetics during the morphological evolution in heteroepitaxial systems [33–36]. Moreover, it has been shown to properly describe the evolution towards equilibrium including realistic anisotropic surface energies [37–39].

Without the loss of generality, we shall focus on the relevant cases of pit-patterned Si(001) surfaces, widely investigated in the literature [8, 10, 14, 30, 40, 41].

The work is organized as follows. In the “Phase-Field Model” section, we briefly illustrate the phase-field model used to describe the evolution by surface diffusion including anisotropic surface energy. Moreover, we describe how the actual Si Wulff shape is accounted for in the considered approach. In the “Smoothing of Si(001) Pits” section, the expected smoothing of Si(001) pits, driven by the surface-energy reduction, is discussed by considering different initial configurations, outlining the kinetic pathway towards the equilibrium. In the “Mimicking the Shape Change due to Ge Overgrowth” section, an application of the method to a specific case of heteroepitaxial growth that corresponds to the surface-energy-driven shape change when depositing a thin layer of Ge on Si pit is considered. Conclusions and remarks are summarized in the “Conclusions” section.

## Methods

### Phase-Field Model

The phase field model considers a continuous order parameter *φ*, varying between *φ*=1 (solid) and *φ*=0 (vacuum) [31, 32]. The approach is based on an energy functional [37],

1 $$ \begin{aligned} F=&\int_{\Omega} \gamma(\hat{\mathbf{n}}) \left(\frac{\epsilon}{2} |\nabla \varphi|^{2} + \frac{1}{\epsilon}B(\varphi) \right) d\mathbf{r} + \\ &+\int_{\Omega} \frac{\beta}{2\epsilon} \left(-\epsilon\nabla^{2}\varphi+\frac{1}{\epsilon}B'(\varphi)\right)^{2} d\mathbf{r},  \end{aligned}  $$

with $\Omega \in \mathbb {R}^{3}$ the domain of definition of *φ*(**r**) and **r**=(*x*,*y*,*z*). The first term corresponds to the interface energy between phases within the diffuse-interface domain defined by *φ*, i.e., to the surface energy of the solid phase. $\gamma (\hat {\mathbf {n}})$ is the surface energy density, with $\hat {\mathbf {n}}$ the outward-pointing surface normal, and *ε* the thickness of the interface between phases. *B*(*φ*)=18*φ* ^2^(1−*φ*)^2^ is a double-well potential with a minima in *φ*=0 and *φ*=1 as in Ref. [31]. The second term in Eq. (1) is the Willmore regularization that is required in the strong anisotropy regime to avoid the formation of sharp corners [37, 38, 42]. *β* is a parameter corresponding to the corner rounding.

The evolution for *φ* reproduces the diffusion-limited kinetics of surfaces and is given by the degenerate Cahn-Hilliard model, i.e.,

2 $$ \frac{\partial \varphi}{\partial t}= D \nabla \left[ M(\varphi) \nabla \mu \right],   $$

where *μ*=*δ* *F*/*δ* *φ* is the chemical potential, *D* is the diffusion coefficient, and *M*(*φ*)=(36/*ε*)*φ* ^2^(1−*φ*)^2^ is the mobility function restricted to the surface. The equation for *μ* reads

3 $$ \begin{aligned} g(\varphi)\mu = \delta F/ \delta \varphi= &-\epsilon \nabla \cdot \left[\gamma(\hat{\mathbf{n}}) \nabla \varphi \right] + \frac{1}{\epsilon} \gamma(\hat{\mathbf{n}}) B'(\varphi) + \\&-\epsilon \nabla \cdot \left[|\nabla \varphi|^{2} \nabla_{\nabla \varphi} \gamma(\hat{\mathbf{n}}) \right] + \\ &+\beta\left(-\nabla^{2} \kappa + \frac{1}{\epsilon^{2}} B^{\prime\prime}(\varphi) \kappa \right),  \end{aligned}  $$

with *κ*=−*ε*∇^2^ *φ*+(1/*ε*)*B* ^′^(*φ*) and *g*(*φ*)=30*φ* ^2^(1−*φ*)^2^ [33, 37, 38]. The latter is a stabilizing function which ensures second-order convergence in the interface thickness, without affecting the description of material transport via surface diffusion [43, 44]. The profile in the direction perpendicular to the interface at equilibrium is well described by

4 $$ \varphi(\mathbf{r})=\frac{1}{2}\left[1-\tanh \left(\frac{3 d(\mathbf{r})}{\epsilon} \right) \right],   $$

where *d*(**r**) is the signed distance to the center of the interface between phases. This equation is adopted to set the initial condition for *φ* as specified in the following. We refer to the surface of the solid phase as the *φ*∼0.5 isosurface. All the geometrical properties of the considered surface can be derived from *φ*, such as the outward-pointing surface normal $\hat {\mathbf {n}}= - \nabla \varphi / | \nabla \varphi |$.

#### Anisotropic Surface Energy

In order to describe anisotropic surface energies, we considered the definition of the surface energy density, $\gamma (\hat {\mathbf {n}})$, as introduced in [38, 39]:

5 $$ \gamma(\hat{\mathbf{n}})=\gamma_{0} \left(1-\sum_{i}^{N} \alpha_{i} \left(\hat{\mathbf{n}} \cdot \hat{\mathbf{m}}_{i} \right)^{w_{i}} \Theta\left(\hat{\mathbf{n}} \cdot \hat{\mathbf{m}}_{i}\right) \right).   $$

where the preferential orientations $\hat {\mathbf {m}}_{i}$, i.e., the directions along which the surface-energy density has a minimum, can be arbitrarily set along with their relative depths, *α*_*i*_, with respect to *γ*_0_. The parameters *w*_*i*_ control the extension of the regions where $\gamma (\hat {\mathbf {n}})<\gamma _{0}$ around **m**_*i*_ directions, i.e., they are namely the widths of the minima (see also Ref. [38]).

To account for the specific anisotropy of Si crystals, we set the minimum energy directions, **m**_*i*_, corresponding to 〈001〉, 〈113〉, 〈110〉, and 〈111〉 [45]. *α*_*i*_ coefficients, determining the depth of minima, are obtained by [39]

6 $$ \alpha_{i}=1-\left(\frac{\gamma_{i}}{\gamma_{\langle 001\rangle}}\right)\left(1-\alpha_{\langle 001 \rangle}\right),   $$

where *α*_〈001〉_=0.15 is set as reference and the various *γ*_*i*_ correspond to the surface energy values of the aforementioned orientations as reported in Ref. [45]. Without the loss of generality, we set *γ*_0_=1. Indeed, the ratios of the minima and the strength of the anisotropy can be controlled by the *α*_*i*_ values from Eq. (6) and *α*_〈001〉_, while *γ*_0_ plays the role of a prefactor in Eq. (2), thus affecting only the absolute time scale of the evolution.

The width of the energy minima in Eq. (5) are set to *w*_*i*_=50 for all the minima directions, except for *w*_〈113〉_=100 [39]. According to this definition of the parameters, sharp corners are predicted in the Wulff shape, i.e., the surface-energy anisotropy is “strong” [38, 42, 46]. Therefore, the Willmore regularization is strictly necessary to perform the simulations. The *β* value sets the extension of the rounded region at the corners, which are known to have a radius proportional to $\sqrt {\beta }$ [37]. In order to perform simulations, the length scale set by the rounding at the corner by *β* has to be larger than the resolution of the spatial discretization of the numerical method. However, it is worth mentioning that small facets possibly present in the Wulff shape with an extension in the order of $\sqrt {\beta }$ may result hidden when using too large *β* values as well as small scale faceting involving preferential orientations actually present in the Wulff shape. In this work, we set *β*=0.005. According to the size of the simulation domain, specified in the following, this value allows us to adopt feasible spatial discretization. Moreover, all the preferential orientations entering Eqs. (5) and (6) are reproduced. On the other hand, possible faceting involving smaller scales than ∼0.07 cannot be reproduced due to the extension of the corner rounding.

#### Initial Morphology and Simulation Setup

In order to investigate any morphological evolution by the phase-field model defined in this section, a proper initial condition for *φ* has to be set. We consider here a smooth pit geometry carved in a (001) planar surface, with a reference frame set to $\hat {\mathbf {x}}=\,[\!100]$, $\hat {\mathbf {y}}=\,[\!010]$, and $\hat {\mathbf {z}}=\,[\!001]$. In particular, we consider a circular (001) surface with radius *L* at a height *h*_0_−*H*, smoothly connected to the surrounding (001) planar surface at height *h*_0_. Such a geometry is set as initial condition for *φ* by exploiting Eq. (4) with *d*(**r**) the signed distance from the surface *Γ*(*x*,*y*) defined by

7 $$ \Gamma(x,y)= \left\{ \begin{aligned}h_{0} - & H & \qquad r \leq L \\ h_{0} - & H \exp \left[ -\frac{1}{2}\frac{|\mathbf{s}-\bar{\mathbf{s}}|^{2}}{\sigma^{2}} \right] & \qquad r> L \end{aligned} \right.  $$

with $r=\sqrt {x^{2}+y^{2}}$ and

8 $$ \mathbf{s}=(x,y), \qquad \bar{\mathbf{s}} =\frac{R}{r} (x,y).  $$

*R*=*H*/4*L* is defined as an aspect-ratio parameter, while *σ* is a parameter controlling the extension of the continuous connection between the bottom of the pit and the flat region surrounding it. This parameter is set here to *σ* = *L*/2.

In Fig. 1, the initial condition adopted for *φ* is illustrated. Figure 1 a shows *Γ*(*x*,0) profiles with different values of *R*. Figure 1 b shows the definition of *φ* by means of Eq. (4) in a 3D parallelepiped domain. In particular, this panel shows a cross-section passing through the center of the whole domain. The left part shows the region corresponding to the solid phase, i.e., the region where *φ*>0.5, revealing the surface that corresponds to the initial pit morphology. The right part illustrates the values of *φ* in the entire 3D domain, i.e., in the bulk phases and within the continuous transition between them.

**Fig. 1:** Initial condition for the phase-field model, resembling a smooth pit at the (001) surface of a solid film. **a** *Γ*(*x*,0) profiles from Eq. (7) obtained for different *R* values. **b** Definition of *φ* in the 3D domain adopted for numerical simulations. It is obtained from Eq. (4) with *d*(**r**) the signed distance from *Γ*(*x*,*y*) with *R* = 0.5. On the left, the solid phase where *φ* > 0.5 is shown. On the right, a color map showing *φ* in the 3D domain is reported

Numerical simulations are performed to integrate Eqs. (2) and (3). They are carried out by using the finite element method (FEM) toolbox AMDiS [47, 48], with a semi-implicit integration scheme and mesh refinement at the interface [33, 38, 49]. Periodic boundary conditions are set along $\hat {\mathbf {x}}$ and $\hat {\mathbf {y}}$ directions. No-flux (Neumann) boundary conditions are set at the top and the bottom of the simulation domain along the $\hat {\mathbf {z}}$ direction. The time scale of the evolution is scaled by a factor 1/*D*, which corresponds to set *D*=1. In the following, we refer to the time of simulations in arbitrary units. The size of the pit is arbitrarily set to *L*=1, while the interface thickness is set to *ε*=0.2.

## Results and Discussion

### Smoothing of Si(001) Pits

In this section, we illustrate the results concerning the morphological changes during the evolution of pit-patterned Si(001) substrates. The model described above allows for the description of the specific case of silicon by means of the definition of the anisotropic surface energy as in the “Anisotropic Surface Energy” section. We expect the following results to be valid from a qualitative point of view for any size, provided that the system is large enough to adopt a continuum approach ($\gtrsim 10$ nm) [32] and the shape can be parametrized by the aspect ratio *R* similar to Fig. 1 a. The real length scale can be considered by setting the *L* parameter to the corresponding one in real units, *L* ^r^. The real time scale can then be described by accounting for real values of *D* and *γ*_0_ and multiplying by the *L* ^r^ length, i.e., by scaling by *L* ^r^/*L* with *L* unitary as specified above.

Let us first focus on the first stages of the evolution. The initial condition set by Eq. (7) consists of a profile which does not exhibit any preferential orientation of the surface. When considering the evolution by surface diffusion driven by the reduction of an anisotropic surface energy, a faceting of the initial profile is expected. This is illustrated in Fig. 2 where the faceting of two profiles with *R*=0.25 in Fig. 2 a and *R*=0.5 in Fig. 2 b are reported. A color scale illustrates the values $\gamma (\hat {\mathbf {n}})$ at the surface. This allows to identify the facets as the regions with an almost uniform surface-energy density corresponding to the minima of Eq. (5), bounded by localized regions with high values of $\gamma (\hat {\mathbf {n}})$. According to the initial aspect ratio of the pit, different facets form. For the smaller R, the (001) facet at the bottom is maintained assuming a squared shape. The edges of the pit result bounded by four {113} facets connected by small, triangular-shaped {110} facets. According to the larger aspect ratio, a larger faceted surface is present when considering *R*=0.5, allowing for the appearance of preferential orientations with higher slope with respect to the (001) surface. In particular, the initial shape allows for the presence of {111} facets forming between two {113} facets close to the bottom and to the flat region. In between, wide {110} facets form.

**Fig. 2:** Faceting of the initial profile as defined in the “Initial Morphology and Simulation Setup” section according to surface diffusion and $\gamma (\hat {\mathbf {n}})$ reproducing the surface energy of Si. Two different initial morphologies are considered: **a** *R* = 0.25 and **b** *R* = 0.5. On the faceted morphologies, symbols are adopted to identify the families of facets. The color scale shows the values of $\gamma (\hat {\mathbf {n}})$ at the surface

The results reported in Fig. 2 show the possibility to predict faceted pit morphology according to the aspect ratio or, in general, according to the initial morphology. We now investigate also the long time scale dynamics inspecting the morphological evolution up to equilibrium [38]. This is illustrated in Fig. 3 where we focus on the deepest pit considered so far, i.e., with *R*=0.5, and the main morphological changes are shown. In particular, perspective and top views of the different morphologies obtained during the evolution are reported in Fig. 3 a, b, respectively. In the first stage of this simulation, we observe the disappearance of the steepest {111} facets and the enlargement of neighbouring {113} facets. Then, the latters merge and the shrinkage of {110} facets begins. These are found to disappear at later stages after assuming a triangular shape, giving a square outline to the pit from a top view. Also, {113} facets eventually vanish and a global flattening is achieved. The real time scale obtained in this simulation can be estimated with data from the literature. In particular, we can consider *D* determined by Arrhenius law with prefactor and activation energy from Ref. [50], where also thermal fluctuations are accounted for. *γ*_0_ is set to have $\gamma (\hat {\mathbf {n}})\sim 8.7$ eV/nm^2^ when $\hat {\mathbf {n}}=(001)$ [51] from Eq. (5), that is, *γ*_0_=10.2 eV/nm^2^. The other material-dependent coefficients of surface diffusion [28], i.e., atomic volume and density at the surface, are set to reproduce the case of Si. According to these values, the expected duration of the entire process at high temperature T ∼1100−1200 °C for *L* ^r^ of tens of nanometers is in the order of hours.

**Fig. 3:** Evolution towards the equilibrium for a Si pit having an initial morphology as in Fig. 2b. **a** Perspective view showing the main morphological changes. **b** Top view of the morphologies in panel **a**. The time reported in panel **b** is expressed in arbitrary units. The color scale shows the values of $\gamma (\hat {\mathbf {n}})$ at the surface

Along with the specific morphological changes occurring during the evolution, two main features should be noticed. First, the evolution leads to the expected global flattening of the surface, and this occurs with the gradual disappearance of steep facets replaced by shallower ones. Although this behavior can be inferred just by arguments about energy minimization and lowering of the aspect ratio, it is worth pointing out that the full evolution is provided here, dealing with the presence of similar facets but with different relative sizes. This is in agreement with the fact that the morphologies obtained during the evolution correspond to out-of-equilibrium configurations and define a pathway towards the global energy minimum. Then, despite the expected facets and their energetics are known, the specific morphology at a certain point of the evolution can be described only by accounting for the dynamics and not just by considering global energy minimization [38].

The second important point shown by the results reported in Fig. 3 is about the intermediate stages. When the shape during the evolution approaches a geometry with a depth similar to the initial profile obtained with *R*=0.25, i.e., at *t*∼3.2, the morphology induced by the energy minimization resembles very closely what is reported in Fig. 2 b, even when starting from an initial configuration with a significant difference in the depth (double in this case). This suggests the existence of a common kinetic pathway toward the final flattening, which is reached after the first fast faceting of the initial morphology. This argument is actually confirmed and further illustrated in the plots of Fig. 4. Here, the monotonous energy decay during the evolution after the initial faceting is reported when considering pits with *R* equal to 0.1, 0.25, 0.5, and 0.75 as in Fig. 1 a. In Fig. 4 a, the time scale expressed in arbitrary units is considered. In Fig. 4 b, the same energy changes are reported with a proper shift of the time scale, highlighting the similar energy decay when approaching similar aspect ratios of the structure. $t^{*}_{R}$ is defined as the time at which the planar surface is obtained, i.e., the time at which the global energy minimum is reached, that is different for each simulation as shown in Fig. 4 a. As shown in this plot, the energy decays almost overlap for *R*≤0.5. A very small difference is observed only when considering *R*=0.75, whose energy decay results are still very close to the other curves and differences basically vanish for $t \gtrsim 5.0$. It is worth mentioning that for large deviations from the initial configuration, namely, with *R*≫1, such geometries may evolve differently with different effects on time scales and morphologies [52, 53]. Moreover, topological changes are known to occur in extreme cases, e.g., with very deep trenches, preventing the possibility to reach the global equilibrium with a flat (001) surface [34, 39, 54].

**Fig. 4:** Energy decreasing during the evolution of pit geometries. **a** *F*(*t*) normalized by the energy of the flat (001) surface obtained as final stage of the evolution. Energy decays obtained from the simulations having different *R* for the initial profile, namely, from *R* = 0.1 to *R* = 0.75, are shown. Time is expressed in arbitrary units. **b** Curves as in panel **a** shifted in order to match $t_{R}^{*}$, i.e., the time at which the global flattening of the pit is achieved depending on *R*

The shapes obtained in the simulations reported in these sections are expected to be observed in experiments, in particular when the processing involves conditions close to the thermodynamic limit. Some of the morphologies reported in Fig. 3 actually do correspond to the outline of pit-patterned Si(001) substrates. For instance, a morphology made of a wide (001) surface bounded by narrow {113} facets as in Fig. 3 at *t*∼5.0 are observed when considering pit-patterned Si(001) substrates with an aspect ratio of 0.05<*R*<0.1 as in Ref. [10, 30]. Also, the relative extension of the facets in the aforementioned stage of the simulation of Fig. 3 is very similar to what was reported in these experimental works. This agreement between simulations and experiments further assesses the theoretical description of surface diffusion adopted here. However, we focused on the general features of the process and a more detailed comparison to specific experiments is out of the purpose of the present work.

### Mimicking the Shape Change due to Ge Overgrowth

As mentioned in the introduction, one of the main applications of pit-patterned Si templates is the control of the growth of self-assembled islands [55]. This holds true in particular when considering the positioning of Ge or Si_1 − *c*_Ge_*c*_ islands on Si(001) substrates [6]. With the methodology adopted in the previous section, we can inspect the morphological changes related to the peculiar features of the surface energy. Therefore, by starting from a proper initial configuration resembling the real morphology of a Si pit and accounting for the differences in the surface-energy density expected when depositing another material, we can predict what is the corresponding contribution to morphological changes.

The case study consists here in the overgrowth of Ge over a Si(001) pit-patterned substrate with an aspect ratio close to 0.1. The profile of Fig. 3 at *t*=5.0 is considered as an initial morphology. Then, a surface energy including also a minima along the 〈105〉 directions is set. This definition of $\gamma (\hat {\mathbf {n}})$ mimics the presence of the small-slope most favorite orientation in Ge/Si(001) systems [56–58]. The high stability of {105} facets is due to the interplay between surface reconstruction and strain effects related to the lattice mismatch between the epilayer and the substrate [59–61]. The surface-energy density value which has to be used in Eq. (6) is taken from Ref. [58] in the limit of a thick Ge layer. Notice that other facets that have a surface energy closer to the (001), such as {1 1 10}, are neglected here. As the angles between the 〈105〉 and the [001] directions are very small, *w*_*i*_ parameters larger than the ones adopted before are required to properly describe the energy minima of Eq. (5) [38]. In particular, we set *w*_{105}_=*w*_{001}_=500.

In Fig. 5, the evolution by surface diffusion with the new definition of $\gamma (\hat {\mathbf {n}})$ is reported. Figure 5 a shows the morphological evolution of the surface with a magnification of the *z*-axis by a factor 5. In the first stages, {105} facets form between the {113} facets present in the initial profile. As 〈105〉 orientations have the minimum energy as also illustrated in Fig. 5 b, the corresponding facets extend while {113} facets shrink. At later stages, a pit bounded by {105} facets only form with still a (001) surface at the bottom. From the top view as in Fig. 5 b, the change in the morphology results in a rotation of the outline of the pit by 45°. This is actually observed during the deposition of Ge on Si-patterned substrates in experiments [41] or during the spontaneous growth of pits due to defects or impurities [40]. The formation of {105} facets is also found to act as a favorite nucleation site for further growth of Ge dots [30]. The evolution illustrated in Fig. 5 demonstrates that a change in shape leading to the rotation of the pit outline can be achieved due to surface-energy reduction only. This is expected to be the real situation in close-to-equilibrium conditions, when thermodynamic driving forces are dominated by surface contributions, i.e., for small Ge volumes. Actually, in order to fully describe the process, elasticity effects, intermixing, and the growth of the solid phase must be included [32]. It is also worth mentioning that even shallower Si pits are adopted in experiments, showing facets with normals along {11*n*} directions, with 5<*n*<10 [41] (i.e., {1 1 10} facets). Pit geometry bounded by these facets would lead to a similar evolution, as they correspond to what adopted as initial configuration of Fig. 4 with just a smaller slope with respect to the (001) plane.

**Fig. 5:** Evolution of the profile in Fig. 3 at *t*=5.0, with a definition of the surface energy including 〈105〉 orientations. **a** Surface profiles at representative stages of the evolution towards the formation of a pit bounded by {105} facets only. *z*-axis is magnified by a factor 5. **b** Top view showing the $\gamma (\hat {\mathbf {n}})$ values at the surface. The second and the last stages of panel **a** are reported in the top and bottom part, respectively. Symbols as in Fig. 2 are adopted to identify different families of facets

## Conclusions

In this work, we have used a continuum model based on surface-diffusion to investigate the temporal evolution of pits excavated in a Si(001) substrate. By suitably tackling (strong) surface-energy anisotropy, with a parametrization based on the well-known Si Wulff’s shape, we have predicted typical metastable configurations in agreement with experiments, including the case where deposition of a different material introduces new stable facets. The entire evolution towards the global flattening of the pit has been illustrated, and it is found to follow the same kinetic pathway also when considering pits with different initial depths. We believe that the model can be predictive also for initial configurations strongly deviating from the ones which we have analyzed as examples. As a consequence, the present approach can be useful in designing experiments based on still-unexplored pit shapes. Furthermore, the model is general and can be easily adapted to different substrates upon re-parametrizing the surface energy.
